The article "Sodium Butyrate Attenuated Diabetes-Induced Intestinal Inflammation by Modulating Gut Microbiota" was published in 2022. Journal: Evid Based Complement Alternat Med.

# Sodium Butyrate Attenuated Diabetes-Induced Intestinal Inflammation by Modulating Gut Microbiota

**DOI:** 10.1155/2022/4646245

**Published:** 2022-08-22

**Authors:** Liping Liu, Yuping Chen, Qin Wu, Anmei Shu, Jihu Sun

**Affiliations:** ^1^College of Pharmacy, Jiangsu Vocational College of Medicine, #283 Jiefang South Road, Yancheng 224000, Jiangsu, China; ^2^Department of Basic Medical Science, Jiangsu Vocational College of Medicine, Yancheng 224005, Jiangsu, China; ^3^Medical College, Jiangsu Vocational College of Medicine, #283 Jiefang South Road, Yancheng 224000, Jiangsu, China; ^4^College of Pharmacy, Nanjing University of Chinese Medicine, #138 Xianlin Road, Nanjing 210000, Jiangsu Province, China; ^5^Institute of Biotechnology, Jiangsu Vocational College of Medicine, #283 Jiefang South Road, Yancheng 224000, Jiangsu, China

## Abstract

**Background:**

Diabetes mellitus (DM) continues to be one of the world's most costly and complex metabolic disorders. Accumulating evidence has shown that intestinal dysbiosis and associated inflammation can facilitate the onset and progression of DM. In this work, our goal was to investigate how sodium butyrate (SB) controls the gut microbiota to reduce the intestinal inflammation brought on by diabetes.

**Methods:**

Male KK-Ay mice were randomized into two groups: the DM model group (intragastric administration of 0.9% normal saline) and the SB treatment group (intragastric administration of 1,000 mg/kg/d SB). The C57BL/6J mice were used as the control group (intragastric administration of 0.9% normal saline). These mice were administered via gavage for 8 weeks.

**Results:**

The results revealed that SB-treated mice significantly reduced fasting blood glucose (FBG), body weight, 24 h food and water intake, and improved islet histopathology in DM model mice. SB reduced TNF-*α*, IL-1*β*, and iNOS, whereas it enhanced the expression of the anti-inflammatory Arg-1 marker on intestinal macrophages and the secretion of anti-inflammatory IL-10. Specifically, SB was linked to a marked drop in the expression of the Th17 marker ROR*γ*t and a substantial increase in the expression of the Treg marker Foxp3. SB treatment was associated with significant reductions in the levels of Th17-derived cytokines such as IL-17 and IL-6, whereas anti-inflammatory Treg-derived cytokines such as TGF-*β* were increased. Additionally, the analysis results from 16S rDNA sequencing suggested that SB significantly reversed the variations in intestinal flora distribution and decreased the relative abundance of *Weissella confusa* and *Anaerotruncus colihominis* DSM 17241 at the species level as well as *Leuconostocaceae*, *Streptococcaceae*, and *Christensenellaceae* at the family, genus, and species levels. These distinct florae may serve as a diagnostic biomarker for DM-induced intestinal inflammation. In addition, the heat map of phylum and OTU level revealed a close relationship between DM-induced intestinal inflammation and intestinal microbiota.

**Conclusions:**

The present study suggested that SB may reduce DM-induced intestinal inflammation by regulating the gut microbiota.

## 1. Introduction

Diabetes mellitus (DM) is a chronic low-grade inflammatory, metabolic disease in which patients present with symptoms including insulin resistance and elevated blood glucose levels. DM is one of the primary causes of death, with approximately 451 million cases among adults >18 years old in 2017, and this number is expected to rise to 693 million by 2045 [1, 2]. Growing evidence suggests intestinal dysbiosis and associated inflammation may facilitate DM onset and progression [3–5]. According to the reported studies, the intestinal inflammation observed in db/db mice has been associated with abnormal enteric glucose sensor functionality that results in inaccurate neuronal signaling and a consequent failure to increase hypothalamic NO release [6]. The role of intestinal inflammation as a mediator of DM progression has also been supported by work using mice in which the innate immune receptor toll-like receptor 5 (TLR5) had been knocked out [7, 8]. Moreover, high-fat diet (HFD) consumption is known to cause significant increases in total gut permeability, gastrointestinal inflammation, and oxidative stress. DM is frequently associated with changes in the composition or permeability of the intestinal barrier [9–12]. The reported studies have suggested that discovering novel methods for decreasing intestinal inflammation in DM patients may be a promising option for slowing disease progression or alleviating related symptoms [13]. In addition, accumulating data suggests that gut immunity plays a vital role in regulating glucose homeostasis [14, 15]. In recent decades, it has been revealed that inhibition of colonic pro-inflammatory macrophage infiltration might prevent HFD-induced insulin resistance from relieving DM [16]. These findings suggested that intestinal inflammation and immunological responses may significantly regulate type 2 DM. However, the underlying regulatory mechanism is unknown.

Furthermore, it has been suggested that gut flora disorders accelerate the onset of inflammatory and chronic metabolic diseases [17–20]. Therefore, targeting gut bacteria may be an effective treatment for diabetes-induced intestinal inflammation. It was found that DM patients have been shown to exhibit significantly reduced levels of butyrate-producing bacteria within the gut lumen relative to healthy controls [21], indicating that butyrate may be one crucial mediator of DM progression. Consistent with this hypothesis, previous research suggests that dietary supplementation with butyrate can improve gut integrity and protect against DM in animal model systems [22]. Sodium butyrate (SB) supplementation has also been shown to reduce inflammation and slow disease progression in the db/db murine model of DM [23]. These results suggested that SB could significantly improve DM.

In addition, SB has potential anti-inflammatory properties, affects the intestinal barrier, and plays a role in satiety and oxidative stress [24]. The SB significantly reduced pathological intestinal damage, lowered intestinal inflammation, and repaired intestinal flora disruption in mice with necrotizing enterocolitis (NEC) [25]. Furthermore, SB alters the intestinal flora composition and improves the gut barrier in HFD mice [26]. Additionally, colon cancers in hosts and the composition of the gut flora are also affected by SB. However, the effect of SB on the gut microbiota in treating DM-induced intestinal inflammation is unknown [27]. In this view, the current study used the KK-Ay spontaneous DM mouse model system with features consistent with human T2DM to evaluate the mechanism of action of SB in improving diabetes-induced intestinal inflammation by regulating gut microbiota. The research may offer novel ideas for SB to treat diabetes-induced intestinal inflammation from the perspective of new mechanism exploration.

## 2. Materials and Methods

### 2.1. Materials

Sodium butyrate (Figure 1(a); HPLC ≥ 98.5% purity) was obtained from Sigma-Aldrich (Shanghai) Trading Co. Ltd. (China). TNF-*α*, IL-1*β*, IL-6, IL-10, TGF-*β*, and IL-17 assay kits were purchased from Shanghai Enzyme-linked Biotechnology Co. Ltd. (Shanghai, China). Primary antibodies, including anti-iNOS (Cell Signaling, 13120S), anti-Arg-1 (Cell Signaling, 93668S), anti-ROR gamma(t) (Invitrogen, 14-6988-82), anti-FoxP3 (Beijing Biosynthesis Biotechnology Co. Ltd., Beijing, China, bs-10211R), anti-*β*-actin (Proteintech, 20536-1-AP), and anti-insulin (Abcam, ab181547). Goat anti-rabbit secondary antibodies (cat. no. 10285-1-AP) were obtained from ProteinTech Group, Inc. (Chicago, IL, USA).

### 2.2. Animals

For this study, male KK-Ay (14–15 weeks old, 38–42 g) and C57BL/6J (14–15 weeks old, 18–22 g) mice were purchased from Beijing Huafukang Bioscience Co. Inc. (China; license no. SCXK Beijing 2014–0004) and placed in a standard breeding condition (12 h light/dark cycle; 25 ± 1°C; 55 ± 5% relative humidity).

Before the trial, these experimental mice received two weeks of adapted feeding. The Nanjing University of Chinese Medicine's Animal Ethics Committee approved the current study (approval no. ACU-13 (20161011)).

### 2.3. Experimental Design

KK-Ay mice were fed a high-fat, high-sugar diet for 8 weeks, and C57BL/6J mice were fed a standard chow diet for 8 weeks. Male KK-Ay mice were randomized into 2 groups (*n* = 6/group): the DM model group (intragastric administration of 0.9% normal saline) and the SB treatment group (intragastric administration of 1,000 mg/kg/d SB), while the C57BL/6J mice as the control group (intragastric administration of 0.9% normal saline). For 8 weeks, the treatment was applied orally to the mice. Treated animals were orally administered SB or an equivalent volume of saline for 8 weeks. Control mice were fed a standard chow diet during this period, whereas all other animals were fed an HFD (60.5% standard chow, 24% lard, 10% sugar, 0.2% cholesterol, and 5% egg yolk powder). After 4 and 8 weeks, we measured FBG in all of the above mice using blood collected from the tail vein after a 12 h fast. Before sacrificing study animals, we collected blood samples in heparin-coated tubes. Serum was collected by spinning these tubes for 20 minutes at 3,000 rpm at 4°C before storage at −20°C. Following blood collection, animals were sacrificed, and islet tissue samples were isolated and fixed using 10% formalin. They were then stored at 4°C before use. Colon samples were additionally collected from these animals, were rinsed using a saline solution, and were stored at −80°C.

### 2.4. Histopathological Evaluation

Islet tissue sections were fixed in 10% formalin, embedded in paraffin, sliced up 5 *μ*m sections, and stained with hematoxylin and eosin. Then, islet histology was assessed using a microscope (400×); ImageJ is used to measure the islet area.

### 2.5. Cytokine Level Measurements

TNF-*α*, IL-6, IL-1*β*, TGF-*β*, IL-17, and IL-10 levels in colon samples were assessed via ELISA based on provided instructions. Briefly, the samples were exposed to primary antibodies for an hour in a 96-well plate. Next, the wells were washed 5 times, and 100 *μ*L of the chromogenic substrate was added for 15 minutes at 37°C. Then the absorbance was measured at 450 nm within 15 minutes of adding 50 *μ*L of stop solution to each well.

### 2.6. Western Blotting

Samples of murine colon tissue were collected, homogenized using RIPA buffer containing protease inhibitors, and spun for 20 minutes at 12,000 × *g* at 4°C. A BCA kit was then used to assess the amount of protein in each sample, after which 40 *μ*g of protein per sample was separated via 10% SDS-PAGE and transferred to methanol-activated PVDF membranes. Next, 5% BSA was used to block these membranes for 2 h, and the membranes were incubated overnight with antibodies specific for iNOS, Arg-1, ROR gamma(t), and FoxP3 (all 1:1,000 in 5% BSA) at 4°C. Then the blots were washed thrice using TBST, followed by 2 h incubation with the HRP-linked secondary antibody (1:10,000). After additional washes, the blots were visualized using an enhanced chemiluminescence reagent. *β*-Actin, as a normalization control and ImageJ software, was used to assess band densitometry.

### 2.7. Extraction and PCR Amplification of Fecal DNA

The E.Z.N.A.® soil DNA kit (mega Bio-tek, Norcross, GA, United States) was used to collect fecal microbial DNA. The purity of the DNA was assessed using 1% agarose gel electrophoresis, while the concentration of DNA was determined through a UV-vis spectrophotometer (NanoDrop 2000, Thermo Scientific, Wilmington, USA). Next, the V3-V4 hypervariable regions of the bacterial 16S rDNA gene were amplified by PCR using primer 338F (5′-ACTCCTACGGGAGGCAGCAG-3′).

### 2.8. Illumina Miseq Sequencing and Bioinformatics Analysis

PCR products were extracted from a 2% agarose gel and further purified using the AxyPrep DNA Gel Extraction Kit (Axygen Biosciences, Union City, CA, USA), followed by quantification using the Quantifluor-ST system (Promega, USA). The pure amplified fragments were assembled into a PE2*∗*300 library using the standard operating protocols for the Illumina MiSeq platform (Illumina, San Diego, USA). Raw readings were stored in the NCBI Sequence Readings archive database. Illumina double-terminal reads were joined, filtered, and then conducted by the Quantifluor-ST software package. Then the sequences with ≥97% similarity were allocated to the same operational taxon (OTU). The typical sequences of each OTU were filtered out, and the differences between the dominating species were then examined.

### 2.9. Statistical Analysis

Data are means ± SD and were compared via one-way ANOVAs with Tukey's post hoc test. SPSS 22.0 was used for statistical analysis, and *P* < 0.05 was the significance threshold. To demonstrate the relationship between various flora, FBG, and intestinal inflammatory cytokines, SPSS determined Pearson's correlation coefficient. The differential flora and the above parameters were plotted on a heat map using Pearson's correlation coefficient through GraphPad software.

## 3. Results

### 3.1. SB Treatment Improves Common Symptoms in DM Model Mice

After 0, 4, and 8 weeks of body weight, 24 h water, food intake, and FBG values, all experimental animals were measured. The body weight, 24-hour food and water consumption, and FBG levels of DM model mice were significantly higher than those of control mice. In contrast, the same variables in animals treated with SB were substantially lower than those in DM model mice (Figures 1(b)–1(e)).

### 3.2. SB Treatment Improves Islet Histopathology in DM Model Mice

We analyzed the islet area to assess how SB treatment affected islet histopathology in DM model mice. Islet area was significantly reduced in DM model animals relative to controls (Figure 2; *P* < 0.05), and SB treatment was associated with significant increases in islet area relative to DM model mice (*P* < 0.05).

### 3.3. SB Treatment Alleviates Intestinal Inflammation in DM Model Mice

To assess the impact of SB on intestinal inflammation in DM model mice, we evaluated TNF-*α*, IL-*β*, IL-6, IL-17, IL-10, and TGF-*β* levels in colon samples from these animals. Relative to controls, DM model animals exhibited significantly increased levels of pro-inflammatory factors such as TNF-*α*, IL-*β*, IL-6, and IL-17, as well as significantly reduced levels of anti-inflammatory cytokines such as IL-10 and TGF-*β* (Figure 3; *P* < 0.05). SB treatment was associated with significant reductions in TNF-*α*, IL-*β*, IL-6, and IL-17 levels, as well as with substantial increases in IL-10 and TGF-*β* levels in treated mice relative to those in the DM group (*P* < 0.05).

### 3.4. SB Promotes an Anti-Inflammatory Intestinal Microenvironment in DM Model Mice

Staining for crucial marker proteins, such as iNOS and Arg-1, expressed by macrophages; ROR*γ*t, expressed by Th17 cells; and Foxp3, which Tregs express, allowed researchers to determine how SB affected the anti-inflammatory microenvironment in the intestines of DM model mice. Relative to control animals, DM model animals exhibited elevated expression of pro-inflammatory iNOS in intestinal macrophages and ROR*γ*t^+^ Th17 cells, while levels of anti-inflammatory Arg-1 and Foxp3^+^ Tregs were decreased in these mice (Figure 4; *P* < 0.05).

### 3.5. SB Treatment Modulates the Imbalance of Intestinal Flora in DM Model Mice

Herein, the regulating effect of SB on the DM-associated alteration of intestinal flora was examined using 16S rDNA sequencing. The Shannon index was used to determine intestinal flora's alpha diversity (*α*-diversity). The DM mice model demonstrated a considerably lower Shannon index than controls. The Shannon index's dynamic variations revealed that intestinal flora's abundance was significantly higher in the SB group than in the DM model group (Figure 5(a)). Moreover, PCA indicated that the composition of intestinal flora was different in each group (Figure 5(b)). The findings of the hierarchical clustering tree analysis suggested significant clustering between the control group and the DM model group. Furthermore, the SB treatment group exhibited a better tendency for separation (Figure 5(c)). In addition, LEfSe analysis was carried out to validate bacterial phenotypes with particular variations from phylum to genus to investigate the differences among control, DM model, and SB groups. Moreover, the LDA score (log 10 > 2) demonstrated remarkable alterations in 76 bacterial strains in the 3 groups (Figure 5(d)). The biodiversity of the intestinal flora varied significantly between groups. The control group's differential microbial lineages included 24 different bacterial species, including *Bacteroidales* S24-7 group, *Actinobacteria*, *Bifidobacterium*, *Verrucomicrobiaceae*, *Bifidobacteriales*, and so on. The differential microbial lineages in the DM model group included 36 bacteria such as *Enterobacteriaceae*, *Gammaproteobacteria*, *Enterobacteriales*, *Candidatus Saccharimonas*, *Escherichia Shigella*, and so on. In the SB model group, 16 bacterial species, such as *Odoribacter*, *Rikenellaceae*, *Lachnospiraceae*, *Lachnospiraceae* UCG-001, *Alistipes*, and so on, exhibited the differential microbial lineages. Additionally, the cladogram revealed the predominant bacteria in each category (Figure 5(e)).

### 3.6. SB Treatment Reversed Changes in Microbial Distribution in DM Mice

*Leuconostocaceae*, *Streptococcaceae*, and *Christensenellaceae* were significantly increased in DM model mice relative to controls at the family level. At the same time, SB treatment was associated with a significant decrease relative to DM model mice (Figure 6(a); *P* < 0.05). At the genus level, *Collinsella*, *Weissella*, *Streptococcus*, and Family XIII AD3011 group were substantially more prevalent in DM model mice compared to controls, while SB therapy was linked to a significantly lower prevalence when compared to DM model mice (Figure 6(b); *P* < 0.05). Interestingly, 2 of the 3 groups among the 76 microorganisms were significantly different, including *Weissella confusa* (*Weissella*) and *Anaerotruncus colihominis* DSM 17241 (*Anaerotruncus*). Remarkably, *Weissella confusa* and *Anaerotruncus colihominis* DSM 17241 were increased dramatically in DM model mice relative to controls, while SB treatment was associated with a significant decrease relative to DM model mice (Figure 6(c); *P* < 0.05). Given these results, SB restored the alterations in the underlined microorganisms' distribution and suggested that they could serve as novel biomarkers for identifying intestinal inflammation induced by diabetes.

### 3.7. Correlation Analysis between Differential Flora and Diabetes-Induced Intestinal Inflammation

The relationship between intestinal flora, FBG, intestinal inflammatory cytokines, diabetes-related intestinal inflammation, and intestinal flora was examined using heat map analysis. In these heat maps, the more color is away from blue, the more negatively associated the two parameters are, while the more color is away from red, the more positively correlated the two parameters are. As shown in Figure 7(a), the heat map of phylum level indicated that *Deferribacteres* was positively related to FBG, pro-inflammatory cytokines, including TNF-*α*, IL-1*β*, IL-6, and IL-17, which were negatively associated with IL-10 and TGF-*β*. *Saccharibacteria* was positively related to pro-inflammatory cytokines, that is, TNF-*α*, IL-1*β*, IL-6, and IL-17, and negatively related to TGF-*β*. According to the heat map of OTU level (Figure 7(b)), FBG was negatively associated with *Akkermansia*, *Bacteroidaceae*, and the *Bacteroidales* S24-7 group. Furthermore, *Akkermansia* and *Bacteroidales* S24-7 group were negatively associated with TNF-*α*. In addition, *Lactobacillaceae* and *Lachnospiraceae* NK4A136 group were positively correlated to IL-6, while *Akkermansia* and *Bacteroidales* S24-7 group were negatively related to IL-6. *Lachnospiraceae* NK4A136 group was utterly associated with IL-17, while *Akkermansia* and *Bacteroidales* S24-7 group were negatively related to IL-17. IL-10 was positively correlated with *Akkermansia*, the *Bacteroidales* S24-7 group, and *Bacteroides*, while IL-10 was negatively correlated with the *Lachnospiraceae* NK4A136 group. Consequently, *Akkermansia*, *Bacteroides*, and the S24-7 group of bacteria positively correlated with TGF-*β*.

## 4. Discussion

DM is a group of metabolic diseases characterized by chronic hyperglycemia resulting from defects in insulin secretion, insulin action, or both. Furthermore, it affects 422 million adults across the globe, which is ∼8.5% of the world's population [5, 28, 29]. Several studies suggest that gut dysfunction can lead to diabetes by affecting glucose metabolism, triggering immunological responses, and increasing insulin resistance and low-grade inflammation [30]. According to a recent study, STZ increased pathological damage to the small intestine. This study indicated that high glucose toxicity might cause intestinal epithelium injury, and diabetic mice exhibited a significant drop in the expression of MFG-E8 and an increase in the expression of p-MLKL and HMGB1 in the ileum. The underlined data suggest intestinal inflammation plays a crucial role in DM [31]. Another study found that hyperglycemia could drive intestinal epithelial barrier function by interfering with intestinal epithelial cells in diabetic mice, contributing to the spread of irritating microbial metabolites throughout the body and enhancing the spread of intestinal infections [32].

Furthermore, several studies suggest that gut microbiota plays a crucial role in regulating DM. It has also been found that the low-grade inflammation in DM may be caused by changes in the intestinal flora [33]. These findings suggested that targeting intestinal inflammation and gut microbiota might be potential approaches to treating diabetes. This study also validated the significance of intestinal inflammation and gut microbiota in KK-Ay diabetic mice. We showed a significant link between intestinal flora dysfunction and DM-induced intestinal inflammation.

The KK-Ay spontaneous DM model was employed in this study to assess the impact of intestinal inflammation and gut microbiota on DM development. KK-Ay mice experienced typical DM symptoms such as polyphagia, polydipsia, weight loss, and elevated FBG levels, which were associated with decreased islet area. This was in line with the fact that people with DM frequently exhibit symptoms, including high blood glucose [34]. Significant intestinal inflammation was also observed in DM model mice, accompanied by increased pro-inflammatory cytokines and decreased anti-inflammatory cytokines. Moreover, DM model mice exhibited elevated pro-inflammatory iNOS in intestinal macrophages and ROR*γ*t + Th17 cells, while anti-inflammatory Arg-1 and Foxp3+ Tregs decreased levels. The underlined data suggested that pro-inflammatory macrophages and Th17 cells significantly regulate DM-induced intestinal inflammation, which was consistent with the previous studies [31–33]. 16S rDNA sequencing of fecal intestinal flora revealed that DM model mice exhibited a significant disruption in the intestinal flora. The results of Shannon indexes demonstrated that the abundance and diversity of intestinal flora were dramatically decreased in DM model mice.

Interestingly, the LDA score (log 10 > 2) revealed that the distinct microbial lineages in the DM model group comprised 36 bacteria, including *Enterobacteriaceae*, *Gammaproteobacteria*, *Enterobacteriales*, *Candidatus saccharimonas*, *Escherichia Shigella*, and so on. These characteristic florae may serve as potential markers for diagnosing DM. Substantial evidence has shown that gut microbiota was crucial in regulating DM. Recent studies have reported that *Deferribacteres* [35, 36] and *Saccharibacteria* [37, 38] at the phylum level were significantly increased in DM, suggesting that *Deferribacteres* and *Saccharibacteria* may play a crucial role in regulating DM development. Interestingly, the correlation analysis of gut microbiota with diabetes-induced intestinal inflammation showed that *Deferribacteres* were positively related to FBG, pro-inflammatory cytokines such as TNF-*α*, IL-1*β*, IL-6, and IL-17, which were negatively associated with IL-10 and TGF-*β*. Furthermore, *Saccharibacteria* was positively related to the pro-inflammatory cytokine such as TNF-*α*, IL-1*β*, IL-6, and IL-17 and negatively related to TGF-*β*. According to our preliminary findings, *Deferribacteres* and *Saccharibacteria* may significantly contribute to triggering intestinal inflammation and driving the onset of DM. Additionally, the correlation analysis between the OTU heat map and intestinal inflammation revealed a significant relationship between gut microbiota, intestinal inflammation, and DM. In contrast to *Akkermansia*, *Bacteroidaceae*, and the *Bacteroidales* S24-7 group, *Escherichia Shigella* showed a positive correlation with FBG on the heat map of OTU level. Moreover, *Akkermansia* and *Bacteroidales* S24-7 group were negatively correlated to TNF-*α*. *Lactobacillaceae* and *Lachnospiraceae* NK4A136 group were positively correlated to IL-6, while *Akkermansia* and *Bacteroidales* S24-7 group were negatively related to IL-6. *Lachnospiraceae* NK4A136 group was utterly associated with IL-17, while *Akkermansia* and *Bacteroidales* S24-7 group were negatively related to IL-17. *Akkermansia*, *Bacteroidales* S24-7 group, and *Bacteroides* were positively related to IL-10, while the *Lachnospiraceae* NK4A136 group was negatively associated with IL-10. *Bacteroidales* S24-7 group, *Bacteroides*, and *Akkermansia* were positively correlated to TGF-*β*. These distinct florae could serve as a biomarker for diagnosing intestinal inflammation caused by diabetes.

Butyrate is considered the most potent SCFA for treating DM, even though it accounts for just 15% of total SCFAs [39]. Fasting blood glucose and free fatty acid levels were inversely related to circulating butyrate levels. Once butyrate concentrations rose above physiological levels, butyrate was shown to have anti-inflammatory effects [40]. NaB could improve T2DM development in db/db mice by promoting glycogen metabolism in hepatocytes to maintain blood glucose homeostasis through the GPR43-AKT-GSK3 signaling pathway [41]. Besides, SB could also inhibit the PERK-CHOP pathway of endoplasmic reticulum stress (ERS) to improve the diabetic model rats induced by streptozotocin combined with a high-fat diet [42]. In addition to significantly lowering DM, SB also can reduce intestinal inflammation. Butyrate is produced in high quantities in the colon by bacteria. It can inhibit histone deacetylases within intestinal macrophages, suppressing their patterns of pro-inflammatory gene expression in a DSS-induced colitis model [43]. In vitro, SB significantly inhibited 5-Fluorouracil (5-FU) induced inflammatory responses in THP-1 and Caco-2 cells and maintained the integrity of tight junctions in intestinal mucosal epithelial cells [44]. Moreover, SB significantly reduced pathological intestinal damage, attenuated intestinal inflammation, and improved intestinal flora disturbance in NEC mice [25]. This was the first study to evaluate how SB could be used to treat diabetes by lowering intestinal inflammation and increasing the gut microbiota.

The present findings indicated that SB reduced blood glucose levels, increased islet area, and improved signs and symptoms of DM, including polydipsia and polyphagia. Together, these results confirmed the ability of SB to protect against or treat DM. SB may ameliorate DM by improving intestinal inflammation. We also found that SB treatment significantly reduced pro-inflammatory iNOS expression and promoted anti-inflammatory Arg-1 expression in the intestinal macrophages of treated animals. In line with these results, SB treatment was associated with significant reductions in TNF-*α* and IL-*β* levels. It increased IL-10 levels, further emphasizing the ability of this metabolite to promote an anti-inflammatory microenvironment within the gastrointestinal tract. SB treatment was also associated with decreases in the expression of ROR*γ*t, a marker of pro-inflammatory Th17 cells responsible for producing inflammatory factors such as IL-6 and IL-17, both of which were decreased in samples from SB-treated DM model animals. The expression of the Treg-associated transcription factor FoxP3 was also increased in animals treated with DM. This increase coincided with increases in levels of the Treg-associated anti-inflammatory cytokine TGF-*β*. The results suggested that SB might ameliorate diabetes-induced intestinal inflammation via suppressing intestinal macrophage-mediated inflammation. Also, further modulating the Treg/Th17 balance to promote an anti-inflammatory intestinal microenvironment.

SB significantly reduced the abundance of *Leuconostocaceae*, *Streptococcaceae*, and *Christensenellaceae* in the DM mice at the family level. This was consistent with the enrichment of *Leuconostocaceae* [45, 46], *Streptococcaceae* [47, 48], and *Christensenellaceae* [49] in the pathological state of diabetes reported in the previous literature. These results suggested that SB may target *Leuconostocaceae*, *Streptococcaceae*, and *Christensenellaceae* at the family level to ameliorate diabetes-induced intestinal inflammation. In the DM mice, SB considerably decreased the genus level abundance of *Collinsella*, *Weissella*, Family XIII AD3011 group, and *Streptococcus*. Additionally, *Weissella confusa* and *Anaerotruncus colihominis* DSM 17241 were significantly reduced by SB at the species level. This was consistent with the enrichment of *Collinsella* [50, 51], *Weissella* genus [45] and its species *Weissella confusa* [52], and *Anaerotruncus colihominis* DSM 17241 [52] in the pathological state of diabetes reported in the previous literature. These results also suggested that SB may target *Collinsella*, *Weissella*, *Streptococcus*, and Family XIII AD3011 group at the genus level and *Weissella confusa* and *Anaerotruncus colihominis* DSM 17241 at the species level to contribute to alleviating diabetes-induced intestinal inflammation. Moreover, the heat map correlation analysis between phylum or OTU level and intestinal inflammation further indicated that gut microbiota and intestinal inflammation played a crucial role in driving DM. These results suggested that SB may reduce diabetes-induced intestinal inflammation via modulating gut microbiota. However, further research is needed to extensively evaluate how SB reduces intestinal inflammation caused by diabetes via regulating the underlined differential microbiota indicators.

## Figures and Tables

**Figure 1:** SB improves common symptoms in DM model mice: (a) the chemical structure of SB, (b) FBG level, (c) body weight, (d) 24 h food intake, and (e) 24 h water intake. *n* = 6/group; ^*∗∗*^*P* < 0.01 vs. control and ^##^*P* < 0.01 vs. DM group.

**Figure 2:** SB treatment was associated with significant improvements in islet histology in DM model mice. Following 8-week treatment with SB, islet histology was assessed in DM model mice and control animals. Islet area was significantly reduced in DM model animals relative to controls, whereas SB treatment was associated with significant increases in islet area relative to DM model mice. *n* = 6/group; ^*∗∗*^*P* < 0.01 vs. control and ^##^*P* < 0.01 vs. DM group.

**Figure 3:** SB treatment was associated with reductions in intestinal inflammation in DM model mice. Upon experimental termination, levels of intestinal (a) TNF-*α*, (b) IL-1*β*, (c) IL-6, (d) IL-17, (e) IL-10, and (f) TGF-*β* were measured. *n* = 6/group; ^*∗∗*^*P* < 0.01 vs. control and ^##^*P* < 0.01 vs. DM group.

**Figure 4:** SB treatment promoted an anti-inflammatory state in the intestines of DM model mice. Western blotting was used to assess (a) the Arg-1/*β*-actin ratio, (b) the iNOS/*β*-actin ratio, (c) the Foxp3/*β*-actin ratio, and (d) the ROR*γ*t/*β*-actin ratio in the intestines of mice in the indicated groups. The number of repetitions in each group of western blotting is 3 ^*∗∗*^*P* < 0.01 vs. control and ^##^*P* < 0.01 vs. DM group.

**Figure 5:** The effect of SB on the intestinal flora imbalance of a DM mouse model. (a) Shannon index chart. (b) PCA chart. (c) Hieratical cluster tree. (d) The LDA scores (log 10 > 2) of the microbial taxa significantly affected different groups acquired by LDA analysis. The bar graph represents the LDA score by the horizontal axis, and the vertical axis shows the significantly distinct groups. The greater the difference, the longer the bar. To display the variations for each sample, bar charts are arranged according to scores. (e) Taxonomic cladogram obtained with LEfSe. Differences are displayed in the color of the most abundant class (red for the control group, blue for the DM model group, and green for the SB group). Each circle's diameter is proportional to the taxon's abundance. *n* = 6/group; ^*∗∗*^*P* < 0.01 vs. control and ^##^*P* < 0.01 vs. DM group.

**Figure 6:** Effect of SB on significantly altered gut flora's relative abundance. (a) Differential flora at the family level, a stands for *Leuconostocaceae*, b stands for *Streptococcaceae*, and c stands for *Christensenellaceae*. (b) Differential flora at the genus level, a stands for *Collinsella*, b stands for *Weissella*, c stands for *Streptococcus*, and d stands for Family XIII AD3011 group. (c) Differential flora at the species level, a stands for *Weissella confusa* and b stands for *Anaerotruncus colihominis* DSM 17241. *n* = 6/group; ^*∗∗*^*P* < 0.01 vs. control and ^##^*P* < 0.01 vs. DM group.

**Figure 7:** Correlation analysis between differential flora and diabetes-induced intestinal inflammation: (a) the heat map depicts the relationship between changes in the intestinal flora and the variations in FBG, TNF-*α*, IL-1*β*, IL-6, IL-17, IL-10, and TGF-*β* at the phylum level and (b) the heat map of the correlation between the alterations in the intestinal flora and the alterations in FBG, TNF-*α*, IL-1*β*, IL-6, IL-17, IL-10, and TGF-*β* at the OTU level. *n* = 6/group; ^*∗∗*^*P* < 0.01 and ^∗^*P* < 0.05.

## Data Availability

The data used to support the findings of this study are available from the corresponding author upon request.
